This article has been retracted.

# Diagnostic Value of Abdominal B-Ultrasound for Congenital Heart Disease Complicated with Extracardiac Malformation in the Second Trimester of Pregnancy

**DOI:** 10.1155/2022/6967655

**Published:** 2022-07-07

**Authors:** Yanming Deng, Lili Zhan, Zhouli Yu, Jianfang Wan

**Affiliations:** ^1^Department of Ultrasound Medicine, Shanghai Pudong Hospital, Fudan University Pudong Medical Center, Shanghai, China; ^2^Department of Ultrasound, The Affiliated Suzhou Science & Technology Town Hospital of Nanjing Medical University, Suzhou, China; ^3^Department of Outpatient Clinics, Shanghai Pudong Hospital, Fudan University Pudong Medical Center, Shanghai, China

## Abstract

**Objective:**

To explore the diagnostic value of abdominal B-ultrasound in the diagnosis of congenital heart disease complicated with extracardiac malformations in the second trimester of pregnancy.

**Methods:**

50 pregnant women with congenital cardiac malformations and extracardiac malformations diagnosed in our hospital from 2015 to 2019 were retrospectively analyzed. The diagnostic results and the types of congenital heart disease complicated with extracardiac malformations were compared to analyze the diagnostic value of abdominal B-ultrasound.

**Results:**

In the diagnosis of 50 fetuses with congenital heart disease and extracardiac malformation, the tetralogy of Fallot syndrome accounts for the largest proportion. Abdominal B-ultrasound in the second trimester was associated with a higher detection rate of fetal heart malformation (72%) versus in the third trimester (40%) (*P* < 0.05). The single atrium and single ventricle had the highest diagnostic accuracy of fetal congenital heart malformation in the second trimester. The highest success rate of detection at different gestational weeks was observed at the 14th gestational week (*P* < 0.05). Four-chamber cardiac section (4CV) had the lowest diagnostic accuracy (62%) for cardiac malformations, and the 4CV + three-vessel-trachea plane (3VVT) had the highest diagnostic accuracy (90%) for cardiac malformations.

**Conclusion:**

Abdominal B-ultrasound features a high diagnostic value for congenital heart disease complicated with extracardiac malformations in the second trimester of pregnancy, and the second trimester is the optimal detection timing with the highest detection accuracy.

## 1. Introduction

Fetal congenital heart disease is a common pediatric disease and is mainly caused by a developmental defect or arrest of development in the maternal body. It is a serious fetal malformation and is a major cause of death in children [1–3]. Congenital heart disease may develop either alone or jointly with other defects of the fetus. Studies have shown that 20%–30% of fetuses with heart defects died in the womb, 40%–60% exhibited extremely poor long-term survival, and only about 0.8% of them survived [4,5], which poses a serious threat to the life safety of fetuses and results in a great economic burden to the society and families [6–8]. Therefore, effective prenatal examinations are of great significance. The diagnosis of congenital cardiac malformations complicated with extracardiac malformations in the fetus during pregnancy check-ups may lead to negative emotions and compromised psychological health of the mother. In this study, traditional Chinese medicine (TCM) emotional care was adopted to alleviate the negative emotions of pregnant women. Emotional fluctuations during pregnancy are associated with dysfunctional disorders in the body and may damage the organs in severe cases. Therefore, adjunctive TCM emotional care facilitates the enhancement of the therapeutic effect [3]. To further study the diagnostic value of abdominal B-ultrasound in congenital heart disease complicated with extracardiac malformations in the second trimester, the medical data of 50 pregnant women with congenital heart malformation complicated with extracardiac malformations in our hospital from 2015 to 2019 were retrospectively analyzed.

## 2. Data and Methods

### 2.1. General Data

A retrospective analysis was conducted on 50 pregnant women with congenital heart malformation combined with extracardiac malformations in our hospital from 2015 to 2019. The pregnant women were aged from 21 to 32 years, with an average age of 26.39 ± 1.71 years, including 29 primiparas and 21 multiparas. Pregnant women received pregnancy check-ups in our hospital at a gestational week of 13–26 weeks, with an average gestational week of 23.0 ± 1.2 weeks. 25 of these 50 pregnant women were randomly selected to receive examination in the third trimester, and the diagnostic accuracy of the examinations performed in the second trimester and the third trimester was compared.

### 2.2. Inclusion and Exclusion Criteria

Inclusion criteria are as follows: the pregnant women with single pregnancy and complete imaging and clinical data and who provided written informed consent were included. This study was approved by the Ethics Committee of Shanghai Pudong Hospital, no. PD9087771.

Exclusion criteria are as follows: pregnant women with contraindications related to B-ultrasound; with a family history of genetic diseases; with acute infection, abnormal amniotic fluid, and other pregnancy diseases were excluded.

### 2.3. Methods

Routine examinations were performed using systematic abdominal B-ultrasound (manufacturer: Jiangsu Jiahua Electronic Equipment Co. Ltd.; equipment model: JH-3212). The fetal anatomy, including cranial, spinal, thoracic, abdominal, and limb structures, was observed in cross-sectional and sagittal views, and the fetal peripheral blood flow and fetal nuchal translucency thickness were measured. Fetal edema and fetal cervical lymphoedema were excluded from this group of fetal anomalies. Subsequently, biological indicators including fetal head circumference, abdominal circumference, and biparietal diameter were examined [9–11]. Prenatal examinations were performed in strict accordance with the detection instruction of B-ultrasound. Segmental examinations were carried out on fetal heart and blood vessels, including fetal ventricular position, the connection between atria and ventricles, four-chamber tangent plane, and fetal atrial size. [12–14]. During the examination, the pregnant woman was advised to perform appropriate activities before the examination in the event of fetal malposition [15, 16]. A one-year follow-up was performed after the delivery.

The pregnant women received TCM emotional care. (1) Personalized psychological care. In TCM emotional care, the nursing staff provided personalized psychological interventions according to the emotional characteristics of the patients to help them relax and relieve negative emotions. The emotional care was conducted in accordance with the concept of “positive emotions suppress negative emotions,” and the patients were actively communicated and instructed by the nursing staff to maintain a positive psychological status. (2) Establishment of a positive emotional environment. The participants and their families were given health education to enhance their awareness of the disease and relevant precautions, and their families were guided to offer positive encouragement and comfort to the patients.

### 2.4. Observation Indicators

The diagnostic results and the types of congenital heart disease complicated with extracardiac malformations were compared to analyze the diagnostic value of abdominal B-ultrasound was analyzed.

### 2.5. Statistical Analysis

In this study, data analyses were performed using the SPSS21.0 software, and all measurement data are expressed as (mean ± standard deviation) and analyzed using the *T*-test. All the counting data are expressed as (*n*, %) and analyzed using the chi-square test. The difference between the two groups was considered statistically significant at *P* < 0.05.

## 3. Results

### 3.1. Pathological Diagnosis

Pathological diagnosis showed there were 50 fetuses with congenital heart disease complicated with extracardiac malformation, among which the tetralogy of Fallot had the highest proportion, as shown in Table 1. Individual B-ultrasound images of cardiac malformation are shown in Figure 1.

### 3.2. Examination Results of Different Trimesters

Abdominal B-ultrasound in the second trimester was associated with a higher detection rate of fetal heart malformation (72%) versus in the third trimester (40%) (*P* < 0.05) (Table 2).

### 3.3. Diagnostic Accuracy of Different Heart Sections in the Second Trimester

The single atrium and single ventricle had the highest diagnostic accuracy of fetal congenital heart malformation in the second trimester (Table 3).

### 3.4. Diagnostic Success Rate at Different Gestational Weeks

The highest success rate of detection at different gestational weeks was observed at the 14th gestational week (*P* < 0.05) (Table 4).

### 3.5. Diagnostic Accuracy of Cardiac Malformations

Four-chamber cardiac section (4CV) had the lowest diagnostic accuracy (62%) for cardiac malformations, and the 4CV + three-vessel-trachea plane (3VVT) had the highest diagnostic accuracy (90%) for cardiac malformations (Table 5).

## 4. Discussion

Congenital cardiac malformation is one of the common cardiac defects. Statistics have shown that about 42% of neonatal deaths every year are attributed to congenital heart malformations, and the disease has become the main contributor to infant death [17–19]. Most patients with congenital heart malformations are complicated with extracardiac malformations, which seriously compromise the growth and development of fetuses [20–22]. Prenatal routine B-ultrasound is an effective method to detect congenital heart malformations complicated with extracardiac malformations, with high safety and reliability. An abdominal ultrasound allows visualization of the fetal ventricles and arteries, which facilitates an accurate determination of the disease. In the present study, fetal echocardiography was performed on the pregnant women with a gestational week of 20–26 weeks to obtain more accurate information about fetal precocious heart disease. The optimal period for the diagnosis of cardiac anomalies is 20–24 weeks of gestation, during which the size of the heart chambers in fetuses with congenital heart disease is significantly different than that in normal fetuses of the same age. These differences are attributable to changes in specific chamber filling volume and chamber pressure induced by hemodynamic changes. Maternal risk factors have a significant impact on the occurrence of fetal congenital heart disease, and early pregnancy medication and family history of heart disease are independent risk factors for fetal congenital heart disease. The detection of fetal congenital heart disease depends on the image quality of ultrasound in two-dimensional views and the sensitivity of color Doppler. Multiple views, multiple angles, and multiple time phases contribute to avoiding missed diagnosis of fetal congenital heart defects.

In the present study, Abdominal B-ultrasound in the second trimester was associated with a higher detection rate of fetal heart malformation (72%) versus in the third trimester (40%). The second trimester ranges from 13 weeks to 27 weeks of gestation, during which there is more amniotic fluid in the womb and the fetal heart structure can be better identified. Therefore, the second trimester is considered the most effective timing for the detection of fetus cardiac health. Moreover, pathological diagnosis showed there were 50 fetuses with congenital heart disease complicated with extracardiac malformation, among which the tetralogy of Fallot had the highest proportion (32%) and single ventricle accounts for the least (4%). The highest success rate of detection at different gestational weeks was observed at the 14th gestational week (*P* < 0.05). Furthermore, the detection of 4CV + 3VVT yielded the highest diagnostic accuracy (90%) for cardiac malformations. Andrea et al. revealed that [23] the diagnostic accuracy of congenital heart malformation by the detection of a four-chamber cardiac section combined with three-vessel-trachea plane was the highest among all cardiac sections. This conclusion was consistent with the results of the present study, which further proved the reliability of the present research. TCM emotional interventions, guided by TCM theory, use communications and interactions to encourage and instruct the pregnant women to alleviate their negative emotions and improve their mental health.

In conclusion, abdominal B-ultrasound has a high diagnostic value for congenital heart disease complicated with extracardiac malformations in the second trimester, and the second trimester is the optimal detection timing with the highest detection accuracy.

## Figures and Tables

**Figure 1:** The display of abdominal B-ultrasound in heart detection of three fetuses with cardiac malformation. (a) Pulmonary artery stenosis. (b) Ventricular septal defect. (c) Aortic stenosis.

**Table 1:** Diagnosis of 50 fetuses with congenital heart disease complicated with extracardiac malformation (*n*, %).

Type	Number of cases	Complicated with extracardiac malformation	Composition ratio (%)
Tetralogy of fallot	16	No	32
Right ventricular double exit	9	Space septal defect, pulmonary valve stenosis, mirror heart and aortic valve stenosis	18
Endocardial cushion defect	3	No	6
Transposition of great arteries	5	Space septal defect, pulmonary valve stenosis, mitral valve stenosis	10
Persistent arterial trunk	5	Space septal defect	10
Single atrium	3	No	6
Single ventricle	2	No	4
Atrial septal defect	3	No	6
Tricuspid valve downward deformity	4	Ventricular septal defect	8

**Table 2:** Comparison of fetal cardiac malformations during different pregnancies (*n*, %).

Pregnancy	Number of cases	Number of confirmed cases	Abdominal B-scan
Second trimester	25	88% (22/25)	72% (18/25)
Late pregnancy	25	60% (15/25)	40% (10/25)
*X* ^2^		5.094	5.195
*P* value		0.024	0.023

**Table 3:** Comparison of the diagnostic accuracy of fetal congenital heart malformation in the second trimester (*n*, %).

Type	Pathological diagnosis	Abdominal B-ultrasound	Accuracy (%)
Tetralogy of fallot	16	14	87.50
Right ventricular double exit	9	6	66.70
Endocardial cushion defect	3	8	66.70
Transposition of great arteries	5	4	80.00
Persistent arterial trunk	5	4	80.00
Single atrium	3	3	100.00
Single ventricle	2	2	100.00
Atrial septal defect	3	2	66.70
Tricuspid valve downward deformity	4	3	75

**Table 4:** Success rate of abdominal B-ultrasound in detecting various sections of heart at different gestational weeks (*n*, %).

Gestational week	Number of cases	Four-cavity tangential plane	Left ventricular outflow tract section	Right ventricular outflow tract section
10 weeks	50	72% (36/50)	16% (8/50)	14% (7/50)
12 weeks	50	78% (39/50)	20% (10/50)	14% (7/50)
14 weeks	50	92% (46/50)^*∗*^	80% (40/50)^*∗∗*^	76% (38/50)^*∗∗∗*^

13–27 weeks was the second trimester. ^*∗*^Compared with the 14th week and the 10th week, the difference in the success rate of displaying four-cavity tangential plane was statistically significant (*X*^2^ = 6.78; *P* = 0.009). ^*∗∗*^Compared with the 14th week and 10th week, the difference in the success rate of left ventricular outflow tract section display was statistically significant (*X*^2^ = 41.03; *P* = 0). ^*∗∗∗*^Compared with the 14th week and 10th week, the difference of success rate in right ventricular outflow tract section is statistically significant (*X*^2^ = 38.83; *P* = 0).

**Table 5:** Comparison of the diagnosis of cardiac malformation by different cardiac sections (*n*, %).

Ultrasonic section	Number of cases	Number of cases with accurate diagnosis	Diagnostic accuracy (%)
4CV	50	31	62
4CV + (AR-SAV)	50	33	66
4CV + VOYV	50	36	72
4CV + 3VV	50	42	84
4CV + 3VVT	50	45	90

4CV: four-chamber cardiac section; AR-SAV: short axis section of aortic root; VOYV: left and right ventricular outflow tract sections; 3VV: three-vessel plane; 3VVT: three-vessel-trachea plane.

## Data Availability

All the data generated or analyzed during this study are included in this published article.
